The article "Development of an Auxiliary Device for Patellar and Femoral Joint Tangential Axial Radiographic Imaging and a Method for Obtaining an Optimal Radiographic Image Using the Development" was published in 2022. Journal: Appl Bionics Biomech.

# Development of an Auxiliary Device for Patellar and Femoral Joint Tangential Axial Radiographic Imaging and a Method for Obtaining an Optimal Radiographic Image Using the Development

**DOI:** 10.1155/2022/5951285

**Published:** 2022-10-12

**Authors:** Do-Byung Rhee, Hee-June Kim, Deok-Mun Kwon, Jung-Su Kim, Hyun-Woo Choi, Jong-Ki Kim

**Affiliations:** ^1^Department of Biomedical Engineering, School of Medicine, Catholic University of Daegu, Daegu 42472, Republic of Korea; ^2^Department of Orthopaedic Surgery, School of Medicine, Kyungpook National University, Kyungpook National University Hospital, Daegu 41944, Republic of Korea; ^3^Department of Radiologic Technology, Daegu Health College, Daegu 41453, Republic of Korea; ^4^Department of Biomedical Engineering, School of Medicine, Kyungpook National University, Daegu 41566, Republic of Korea

## Abstract

This study evaluated the accuracy of tangential axial radiography of the patellar and femoral joint using an auxiliary device based on three image evaluation criteria, which we named the patellofemoral joint radiography auxiliary device (PJR). To compare the PJR method with conventional radiographic methods, such as Laurin, Merchant, and Settegast, a whole-body phantom (PBU-31) was used and three image evaluation items were set. The radiographic method, the smallest inclination of the patellar and showed the best half lateral image of the patella, is Settegast, and the measurement is 9.40. The second-best PJR measurement is 9.97, and the difference between the two measures is 5.76% (*p* = 0.001). The radiographic method showing the image with the largest distance between the patellar and femoral joint space is PJR which a measurement is 12.35. The second best Merchant measure is 10.55, and the difference between the two measures is 14.54% (*p* = 0.001). The method in which the two bones were well overlapped (i.e., evaluate the distortion of the image by measured as the distance between the femoral trochlear groove and the tibial tuberosity) is the PJR and the measurement is −0.37. The second-best Merchant measure is 3.93, and the difference between the two measures is 91.4% (*p* = 0.001). The Settegast has the image with the smallest inclination of the patella, but the PJR has the image that best describes the patellar–femoral joint and the least distortion of the image. As a result of the comprehensive evaluation, when using PJR, bending the knee by 40° and setting a 140° angle between the long axis of the femur and the long axis of the lower leg were considered to be the most beneficial conditions. Therefore, we propose the use of PJR for tangential axial radiography of the patellar–femoral joint.

The article "Development of an Auxiliary Device for Patellar and Femoral Joint Tangential Axial Radiographic Imaging and a Method for Obtaining an Optimal Radiographic Image Using the Development" was published in 2022. Journal: Appl Bionics Biomech.

## 1. Introduction

Patellar and femoral joint instability describes an elevated risk of dislocation redislocation of the patella. Patellar–femoral joint instability can occur after traumatic patellar dislocation caused by injury to the patellar–femoral ligaments and can be associated with an increased risk of redislocation. Patellar–femoral joint instability can be the result of unphysiological movement of the patella within the trochlear groove (known as maltracking) resulting in recurrent patellar dislocation or subluxation [1] and could cause cartilage damage to the joint surface [2]. Examinations of the patellar–femoral joint are diverse and include physical examination, radiography, computed tomography, magnetic resonance imaging, and arthroscopy. Among these, visual examination and radiography are the first and main examinations performed to diagnose problems, such as patellar fracture, dislocation, and subluxation and knee joint varus–valgus, and malalignment. There are several radiographic methods to assess various diseases of the patellar–femoral joint. In general, X-ray of the knee joint on two planes (anterior–posterior and lateral) and patellar–femoral joint tangential axial radiography and intercondyloid fossa radiography are mainly performed [3, 4]. Tangential axial radiography is advantageous for evaluating wear on the patellar–femoral joint surface, identifying the half-lateral image of the patella, and understanding the relationship between the femur and tibia. Moreover, it is an important radiographic method for determining patellar–femoral joint structure, shape, and damage [5]. Existing radiography methods have caused distinct problems. The Settegast and Hughston methods perform radiography in a prone knee bending position. This method cannot be used to patients with knee flexion contracture or patellar fractures and dislocations. The Laurin method performs radiography by bending the knee in a sitting position, since a patient must directly hold the detector (image receptor) in a sitting position and perform radiographic imaging, there is a risk of shaking and falling from an unstable position. When performing radiographs by the Merchant method, the legs should be placed in the Merchant-specific auxiliary device in the supine position. Both knees should be radiographed twice each, and the position of the femur should be kept horizontal on the examination table. In addition, the problem with radiographic imaging is the overlap of the femoral trochlear groove and the tibial tuberosity, unclear medial and lateral condyle of femur images, overlap of patellar apex, and abnormal patellar–femoral joint images. Therefore, the authors of this study developed a patellofemoral joint radiography auxiliary device (PJR) to directly solve the problems encountered during conventional imaging. The biggest advantage of the PJR method is that a patient can fine-tune the angle of the knee after putting the leg into an auxiliary device in the supine position. The purpose of this study was to compare the PJR method with conventional radiographic methods for tangential axial radiography of the patellar–femoral joint. In addition, radiographic evaluation items were set and used to compare radiographic images and determine the most suitable among the radiographic methods.

The article "Development of an Auxiliary Device for Patellar and Femoral Joint Tangential Axial Radiographic Imaging and a Method for Obtaining an Optimal Radiographic Image Using the Development" was published in 2022. Journal: Appl Bionics Biomech.

## 2. Materials and Methods

### 2.1. Development

PJR, the name of the present invention, effectively fixes the patient's lower leg and enables movement to improve the efficiency of X-ray examination and reduce patient fatigue. In the PJR, rather than directly moving the body of a lying patient, the examiner adjusts the angle by adjusting the wrench provided in the body of the assistive device, enabling easier X-ray examination. The PJR can form a fixing force not only on the patient's thigh but also on the patient's shin, so that more accurate X-ray imaging can be performed. In addition, the device consists of a detector in four steps to adjust the height and the thickness of the patient's thigh and to fix the sides of the thighs to prevent the movement (Figure 1).

### 2.2. Experimental Equipment

The X-ray imaging equipment used in this study was the Digital Radiography X-ray System (Innovision-SH 3D; DK Healthcare Co., Hisar, Haryana, India). For the wireless detector type, a mobile flat panel detector [FXRD-1417NAW model (CsI)] was used. The left leg, including the patellar and patellar–femoral joint, of the whole-body phantom (PBU-31, Kyoto Kagaku Inc., Kyoto, Japan) was used. The back of the patella is composed of urethane-based resin soft tissue (density: 1.06), and the knee joint is assembled with epoxy resin (density: 1.31) and urethane with carbon fiber material.

### 2.3. Experimental Methods

Using PJR, the phantom knee was bent at 70°– 20° by varying the angle at 10° intervals, and the long axes of the femur and lower leg were set at 110°–160°. At this time, the angles of the X-ray tube and detector were positioned to remain perpendicular to the angle of the patella with every change during knee bend at 10° (Figures 2 and 3(a)). Each of the six radiography methods collected 30 images, and a total of 180 images were compared and analyzed. The Houston method is advantageous for patients who cannot bend the knee less than 45°–55°, but it has a large disadvantage of causing distortion in the radiographic image. Radiography in the prone position was performed only by the Settegast method, in which the X-ray tube was set at an angle of 15° toward the patella by bending the phantom's knee to 105° (Figure 3(b)) [6–9]. 30 Settegast images were collected. The Laurin method is a condition in which the knee is bent by 20° and the long axis of the femur and the long axis of the tibia and fibula are set at an angle of 160° (Figure 3(c)) [10, 11]. 30 Laurin images were collected. The Laurin method is contained within the method using PJR. With the Merchant method, the knee was bent at 45°, each leg was placed in a Merchant-specific assist device, the detector was positioned about 30 cm below the knee, and the X-ray tube was positioned at an angle of 30° toward the patella (Figure 3(d)) [12]. 30 Merchant images were collected. The following radiographic settings were the same for all methods: 55 kV, 250 mA, 0.045 s of exposure time, and a source to image receptor distance (SID) of 110 cm (Figure 4).

The article "Development of an Auxiliary Device for Patellar and Femoral Joint Tangential Axial Radiographic Imaging and a Method for Obtaining an Optimal Radiographic Image Using the Development" was published in 2022. Journal: Appl Bionics Biomech.

The radiographic evaluation items are described as follows:

(a) The distance between the line connecting the medial and lateral sides of the patellar and the lowest point of the median ridge of the patella (DMLP), which was measured to evaluate patellar inclination. The smaller the DMLP measurement result, the better. The reason is that the smaller the DMLP result value, the better the half-lateral image with a smaller patellar inclination. When the angle between the long axis of the femur and the lower leg is changed, so does the angle of the patella. As the bending angle increases, both angles of the X-ray tube and detector also increased.

(b) The patellar and femoral joint space distance (DPFG). The larger the DPFG measurement result, the better.

(c) The distance between the femoral trochlear groove and the tibial tuberosity (DFGT), which was measured to evaluate the degree of overlap between the two bones. As a result of DFGT measurement, values near the number 0 are superior (Figure 5). The measured DFGT values were compared with the smallest and largest values to determine how they affect the DPFG and DMLP evaluation results.

### 2.4. Statistical Analysis

The quantitative values of the radiographic images were measured and evaluated using a Picture Archiving Communication System program (Centricity, GE Healthcare, Chicago, IL, USA). For each measured variable, statistical significance was verified by one-way ANOVA using the Statistical Package for the Social Sciences software (SPSS 20.0, IBM SPSS Statistics, Chicago, IL, USA). Using the PJR, the phantom's knee flexion was changed six times at 10° intervals to find the most appropriate radiographic conditions among the measured values, which were then compared with those by the Laurin, Merchant, and Settegast methods using one-way ANOVA. The statistical significance level was set to *p* < 0.05.

The article "Development of an Auxiliary Device for Patellar and Femoral Joint Tangential Axial Radiographic Imaging and a Method for Obtaining an Optimal Radiographic Image Using the Development" was published in 2022. Journal: Appl Bionics Biomech.

## 3. Results

### 3.1. Phantom Experiment Using the PJR

In all experiments, the X-ray tube angle and detector angle settings were made perpendicular to the patellar angle. A summary of the measurement results is shown in Table 1 and Figure 6(a). The following were the findings with each change in the angle of the phantom's knee six times at 10° intervals using PJR: (a) the smallest inclination of the patella based on DMLP evaluation was when the knee was bent at a 20° angle, the angle between the long axis of the femur and the lower leg was 160°; this was the same method as the Laurin method; (b) the largest patellar and femoral joint space based on DPFG evaluation was when the knee was bend at a 40°, the angle between the long axis of the femur and the lower leg was 140°; and (c) the most overlapping value for the distance between the femoral trochlear groove and the tibial tuberosity based on the DFGT assessment was 140° when the knee bent at 40°, the angle between the long axis of the femur and the lower leg.

The difference in the DMLP values between knee flexion by 20°, 160° angle of the long axis of the femur and lower leg and knee flexion by 40°, 140° angle of the long axis of the femur and lower leg was not significantly different at 0.24% (*p* = 1.000). In the DPFG evaluation, the largest patellar and femoral joint space was when the knee was bent at 40°, and the angle between the long axis of the femur and the lower leg was set to 140°. When the knee was bent at 20°, the angle between the long axis of the femur and the lower leg was 160°, and the change in the DPFG value was not significant at 32.94% (*p* = 0.001). In the DFGT evaluation, the most consistent value between the femoral trochlear groove and the tibial tuberosity was when the knee was bent at 40°, the angle between the long axis of the femur and the lower leg was set to 140°. When the knee was bent at 20°, the angle between the long axis of the femur and the lower leg was 160°, and the change in the DFGT value was significantly different at 92.97% (*p* = 0.001; Table 2). As the DFGT measurement value increased, it was confirmed that the patellar–femoral joint gap, which means wear of the patellar articular cartilage, decreased.

### 3.2. Comparison of PJR with the Settegast and Merchant Radiography Methods

The measured values using PJR with the phantom's knee bent at 40° and the angle between the long axis of the femur and the long axis of the lower leg set at 140° were compared with the values measured by the Settegast and Merchant methods. The results of comparisons of all measurements are shown in Table 3 and Figure 6(b).

The article "Development of an Auxiliary Device for Patellar and Femoral Joint Tangential Axial Radiographic Imaging and a Method for Obtaining an Optimal Radiographic Image Using the Development" was published in 2022. Journal: Appl Bionics Biomech.

In the DMLP evaluation, the smallest patellar inclination and best display of the half lateral image of the patella were with the Settegast method, followed by PJR and the Merchant method. The measured DMLP values significantly differed by 5.76% between the Settegast method and PJR; by 5.62% between PJR and the Merchant methods (*p* = 0.001). In the DPFG evaluation, the largest patellar–femoral joint spacing was seen with PJR, followed by the Merchant and the Settegast methods. The measured DPFG values significantly differed by 14.54% between PJR and the Merchant method; by 19.01% between the Settegast and Merchant methods (*p* = 0.001). In the DFGT evaluation, the distance between the femoral trochlear groove and the tibial tuberosity was the most consistent with PJR, followed by the Merchant and the Settegast methods. The measured DFGT values significantly differed by 91.4% between PJR and the Merchant method; by 27.75% between the Settegast and Merchant method (*p* = 0.001). It was confirmed that the patellar–femoral joint space increased as the DFGT measurement value was closer to the number 0.

## 4. Discussion

This study was conducted to find the most suitable tangential axial radiography method for the patellar and patellar–femoral joint by comparing PJR with the conventional radiographic methods. Among the radiographic conditions using PJR was compared with the conventional imaging methods of Settegast and Merchant. In the DMLP evaluation, when the knee of the phantom was bent at 70°–20° at 10° intervals using PJR, the DMLP value decreased as the angle of flexion was increased. This implied that the inclination of the patellar decreased when the knee was extended than when the knee was flexed and that the half-lateral image of the patellar was more accurately displayed with the former. The Laurin method with a knee flexion angle of 20° had the smallest inclination of the patellar and the half-lateral image of the patella showed the best results. But, based on the DFGT results, as the value representing the distance between the femoral trochlear groove and the tibial tuberosity increased to a positive value, the tibial tuberosity invaded the patellar–femoral joint area and resulted in narrowing of the patellar–femoral joint space. On the other hand, as the distance between the femoral trochlear groove and the tibial tuberosity was reduced to a negative value, the inclination of the patellar became larger. In addition, among the radiographic conditions using PJR, 20° knee flexion, which is similar to that in the Laurin method, and 160° angle of the long axis of the femur to the long axis of the lower leg resulted in the largest invasion of the tibial tuberosity to the patellar–femoral joint and the narrowest patellar–femoral joint spacing (Figure 6(a)). Although the Settegast method gave the smallest inclination of the patellar on imaging, it required the largest knee bending angle and may cause further discomfort to a patient with knee pain. When the distance between the femoral trochlear groove and the tibial tuberosity was the largest and the tibial surface invaded the patellar–femoral joint space, the resulting image had the narrowest joint spacing. The reason for the result of the smallest inclination of the patellar with the Settegast method than with the Merchant and PJR methods was thought to be close contact of the patella with the detector in the prone position. The object-to-image receptor distance (OID) between the patella and the detector was the target area for radiographic imaging. If the OID was short, distortion in the radiographic image was reduced. On the other hand, if the OID was increased, the image was enlarged and had a degraded quality, resulting in blurring and low contrast [13–15]. The Merchant method showed the greatest patellar inclination, and the overlap between the patellar–femoral joint space and the femoral trochlear groove and the tibial tuberosity was not as good as the PJR method, but better than the Settegast method. With the results of the DMLP, DPFG, and DFGT evaluations taken together, 40° knee flexion with 140° angle between the long axis of the femur and the long axis of the lower leg was the most beneficial radiographic condition using PJR (Figure 6(b)).

The article "Development of an Auxiliary Device for Patellar and Femoral Joint Tangential Axial Radiographic Imaging and a Method for Obtaining an Optimal Radiographic Image Using the Development" was published in 2022. Journal: Appl Bionics Biomech.

Tangential axial radiography must be performed in order to detect patellar fracture and injury and patellar–femoral joint stenosis and wear and to determine the correlation between the femur and tibia. However, conventional radiography methods have several disadvantages. First, although the Settegast and Hughston methods are relatively frequent in the clinical setting because of the relatively short procedure time, the required prone position and knee flexion may be difficult in patients complaining of pain from patellar fracture or dislocation [3, 16–18]. In the prone position, the patellar area comes into contact with the examination table and a load is applied; this may worsen the pain in the area near the knee and should be avoided [3, 17]. Second, the Laurin and Merchant methods are radiographic methods that can be used to diagnose patellar–femoral joint disease in a sitting or supine position without the need to prone. The Laurin method mainly measures the lateral patellar–femoral angle and checks whether patellar is normally open to the outside. The Laurin method was said to require the smallest bending angle of the knee and was the closest to the actual structure of the patella [10, 11]. However, as the knee bending angle decreases, the distance between the femoral trochlear groove and the tibial tuberosity increases, the tibial surface invades the patellar–femoral joint space, and the gap narrows. Therefore, this is not suitable for viewing minute damages to the patellar–femoral joint. Moreover, the Laurin method necessitates postural instability, because the patient must bend the knee in a sitting position, directly hold the detector, and perform radiography. In addition, in a sitting position, special care is required to avoid radiation exposure to areas other than the patellar–femoral joint [3].

The article "Development of an Auxiliary Device for Patellar and Femoral Joint Tangential Axial Radiographic Imaging and a Method for Obtaining an Optimal Radiographic Image Using the Development" was published in 2022. Journal: Appl Bionics Biomech.

Most of the existing studies on patellar–femoral joint observation determined patellar dislocation and subluxation by measuring the congruence and sulcus angles [15, 19, 20]. To measure this in the Merchant method, the long axis of the femur must be parallel to the surface of the examination table using an auxiliary device. In the Merchant method, each knee is radiographed separately. When both legs are shot simultaneously, one leg may not be fixed and the knee may be adducted or abducted; these may increase the matching angle and distort the image [19]. In addition, when the distance from the source is doubled, the radiation intensity is proportional to the inverse square of the distance, where the radiation level per unit area decreases to 1/4 [21]. In the case of similar SID, as the distance from the source of the X-ray tube to the object part (SOD) increases, the entrance surface dose decreases. Conversely, as the OID becomes closer, the enlargement of the image is prevented [13, 22]. The set OID was about 30 cm for the Merchant method and about 20 cm for PJR (Figure 7). In this research, because the tangential axial radiography method using PJR had 10 cm longer SOD and 10 cm shorter OID, compared with those by the Merchant method, the latter will create more exposure to radiation doses. Comparison of radiation doses in tangential axial radiography of the patellar–femoral joint requires more in-depth experiments. Nevertheless, radiographic imaging using PJR may be a good means of solving some of the shortcomings of the conventional radiographic methods. Specifically, PJR may allow patients to comfortably undergo radiographic imaging in a supine position and may enable a stable position to prevent shaking or distortion of the image at the target site. Compared with the conventional radiographic methods, PJR showed radiographic images in which the patellar–femoral joint space was larger, the gap between the trochlear groove and the tibial tuberosity was consistent, and the half-lateral image of the patella was clearly shown (Figure 8).

The article "Development of an Auxiliary Device for Patellar and Femoral Joint Tangential Axial Radiographic Imaging and a Method for Obtaining an Optimal Radiographic Image Using the Development" was published in 2022. Journal: Appl Bionics Biomech.

One limitation of this study was that the comparison of different patellar–femoral joints among humans was not possible. However, by performing several patellar–femoral joint radiography imaging on the phantom knee joint, we were able to quantify the most optimal patellar and patellar–femoral joint shapes. In the future, studies that measure the shape of several patellar–femoral joint in humans are needed.

## 5. Conclusions

We propose the use of PJR for tangential axial radiography of the patellar and patellar–femoral joint. PJR may provide convenience to patients and images of high diagnostic value. We look forward to its further use in the clinical field in the future.

## Figures and Tables

**Figure 1:** Development of patellofemoral joint radiography auxiliary device (PJR). (a) Structure of the PJR. (b) The form of widening the angle of the PJR. (c) The form of narrowing the angle of the PJR.

**Figure 2:** Set the X-ray tube and detector angles to be perpendicular to the angle of the patella.

**Figure 3:** Patellar tangential axial radiography imaging. (a) Patellar tangential axial projection method using the PJR. (b) Settegast method. (c) Laurin method. (d) Merchant method.

**Figure 4:** A phantom was mounted on the developed body of the PJR, and radiographs were taken in the tangential axial projection.

**Figure 5:** Measurement items ((1) patella, (2) lateral facet of patella, (3) medial facet of patella, (4) the lowest point of the median ridge of the patella, (5) patellofemoral joint space, (6) femoral trochlear groove, (7) lateral trochlear ridge, (8) medial trochlear ridge, and (9) tibial tuberosity).

**Figure 6:** (a) Results of taking radiographic images at 20° to 70° using PJR and changing the knee flexion angle at 10°. (b) A graph comparing the measurement results among PJR, Merchant method, and Settegast method.

**Figure 7:** Fundamental concepts of source to image receptor distance (SID), source to object distance (SOD), and object to image receptor distance (OID).

**Figure 8:** Phantom X-ray images taken by each method ((a) DMLP, (b) DPFG, and (c) DFGT). (a) Method using PJR. (b) Merchant method. (c) Settegast method.

**Table 1:** Results of taking radiographic images at 70° to 20° by changing the knee flexion angle at 10° intervals using Development of patellofemoral joint radiography auxiliary device (PJR).

PJR used		Measures					
Parameters	70°	60°	50°	40°	30°	20°	*p*-Value
Degree of flexion							
Patellar angle	18°	15°	12°	9°	6°	4°	—
X-ray tube angle	108°	105°	102°	99°	96°	94°	—
Detector angle	72°	75°	78°	81°	84°	86°	—
(a) DMLP	11.27 ± 0.16	10.69 ± 0.23	10.24 ± 0.23	9.97 ± 0.15	9.95 ± 0.1	9.95 ± 0.1	0.001
(b) DPFG	11.16 ± 0.71	11.59 ± 0.68	9.41 ± 0.36	12.35 ± 0.67	10.1 ± 0.53	8.28 ± 0.65	0.001
(c) DFGT	−4.14 ± 0.16	−5.47 ± 0.2	−5.75 ± 0.17	−0.37 ± 0.36	2.5 ± 0.32	4.87 ± 0.26	0.001

DMLP = the distance between the line connecting the medial and lateral sides of the patella and the lowest point of the median ridge of the patellar, which was measured to evaluate patellar inclination. DPFG = the patellofemoral joint space distance. DFGT = the distance between the femoral trochlear groove and the tibial tuberosity, which was measured to evaluate the degree of overlap between the two bones.

The article "Development of an Auxiliary Device for Patellar and Femoral Joint Tangential Axial Radiographic Imaging and a Method for Obtaining an Optimal Radiographic Image Using the Development" was published in 2022. Journal: Appl Bionics Biomech.

**Table 2:** Comparison of PJR images taken at 40° and 20° of knee flexion angles.

Comparison between two groups	Measure		
Parameters	40°	20°	*p*-value
Degree of flexion			
Patellar angle	9°	4°	—
X-ray tube angle	99°	94°	—
Detector angle	81°	86°	—
(a) DMLP	9.97 ± 0.15	9.95 ± 0.1	1.000
(b) DPFG	12.35 ± 0.68	8.28 ± 0.65	0.001
(c) DFGT	−0.37 ± 0.36	4.87 ± 0.22	0.001

**Table 3:** Comparison of the measured values by PJR with those of the Merchant and Settegast methods.

Comparison among three groups	Measure			
Parameters	PJR	Merchant	Settegast	
Degree of flexion	40°	45°	105°	*p*-value
Patellar angle	9°	13°	14.5°	—
X-ray tube angle	99°	60°	15°	—
Detector angle	81°	45°	0°	—
(a) DMLP	9.97 ± 0.15	10.57 ± 0.47	9.40 ± 0.47	0.001
(b) DPFG	12.35 ± 0.68	10.55 ± 0.43	8.54 ± 0.65	0.001
(c) DFGT	−0.37 ± 0.36	3.93 ± 0.23	5.42 ± 0.49	0.001

## Data Availability

Data supporting this research article are available from the corresponding author or first author on reasonable request.

## Additional Points

*Preprinted*. Research article posted in preprint Research Square [23].
